# Beneficial Effects of Crocin against Depression via Pituitary Adenylate Cyclase-Activating Polypeptide

**DOI:** 10.1155/2020/3903125

**Published:** 2020-06-24

**Authors:** Linyu Lu, Die Wu, Kai Wang, Juanjuan Tang, Gang Chen

**Affiliations:** ^1^School of Medicine and Holistic Integrative Medicine, Nanjing University of Chinese Medicine, Nanjing 210023, China; ^2^Interdisciplinary Institute for Personalized Medicine in Brain Disorders, and Research Center for Formula and Syndromes, Jinan University, Guangzhou 510632, China; ^3^Co-innovation Center of Neuroregeneration, Nantong University, Nantong, Jiangsu 226001, China

## Abstract

Depression is one of the foremost psychological illness, and the exact mechanism is unclear. Recent studies have reported that the pituitary adenylate cyclase-activating polypeptide (PACAP) signaling pathway is involved in the progression of depression. In the present study, we extracted crocin from the traditional Chinese medicine (TCM), *Gardenia jasminoides* Ellis, to evaluate its antidepressant effect and clarify the underlying mechanism. Here, we established a chronic unpredictable mild stress (CUMS) mouse model to assess whether crocin can improve depression-like behavior in an open field test (OFT), tail suspension test (TST), forced swimming test (FST), and sucrose preference test (SPT). A corticosterone (CORT) model of PC12 was set up to explore the antidepressant mechanism of crocin. We pretreated PC12 cells with crocin for 1 hour and then stimulated the cells with CORT for 24 hours. Cell survival was detected by Hoechst staining and MTT assay. The expression of PACAP, cyclic adenosine monophosphate (cAMP) response element binding protein (CREB), and extracellular regulated protein kinases (ERK) were analyzed by western blotting. PACAP RNAi was used to interfere with PC12 cells to downregulate the content of PACAP. The results showed that crocin (30 mg/kg) significantly reversed the decrease of body weight and elevation of serum CORT, mitigated CUMS induced depression-like behaviors of mice, and crocin (12.5 *μ*mol/L) protected PC12 cells against CORT (200 *μ*mol/L)-induced injury. Furthermore, crocin greatly increased the protein expression of PACAP and phosphorylation of ERK and CREB in the CORT model. PACAP RNAi cancelled the neuroprotective effect of crocin. In conclusion, these results indicated that crocin exerted an antidepressant effect via upregulating PACAP and its downstream ERK and CREB signaling pathways.

## 1. Introduction

The rapid development of society and economy can produce serious stress and adversity, which may lead to depression. Symptoms of depression include chronic low mood, cognitive impairment, and even suicide [1]. It is now a leading cause of disability and a major contributor to the overall global burden of disease [2]. Conventional antidepressants, typically selective serotonin reuptake inhibitors (SSRIs), have limitations in long lag period, nonresponsive subpopulations, and adverse effects [3]. Therefore, it is urgent to find new strategies for more rapid, effective, and safe antidepressant treatment.

Growing evidences indicate that PACAP, a potent neuropeptide, is involved in neuronal regeneration, synapse formation, and neural plasticity in the central nervous system (CNS) [4, 5]. Clinical studies have shown that a genetic variant of the PACAP gene is associated with depression [6]. PACAP knockout (KO) mice showed prolonged immobility in the forced swim test (FST) [7, 8], which suggests that the PACAP signal pathway may be involved in depression pathogenesis. 180 min maternal deprivation of PACAP heterozygous mice on CD1 background upon CVMS (chronic variable mild stress) may be used as a reliable model for major depression [9]. Furthermore, PACAP activates cyclic adenosine monophosphate (cAMP) response element binding protein (CREB) and extracellular regulated protein kinases (ERK) [10]. The ERK-CREB pathway plays a crucial role in depression. It can regulate the growth, proliferation, and differentiation of hippocampal neurons [11]. All these suggest that PACAP may be a novel potential target for depression treatment.

Crocin is one of the main active ingredients extracted from gardenia, a traditional Chinese medicine. Clinical studies have shown that crocin is as effective as imipramine in the treatment of mild to moderate depression [12]. Further, crocin significantly increases the expression of p-CREB, brain-derived neurotrophic factor (BDNF), and vascular endothelial growth factor (VEGF) in the rat hippocampus [13]. Our previous research showed that Yueju pills [14] and gardenia [15] have antidepressant effects, with gardenia yellow pigment (GYP, a collection of compounds with shared structure of crocin) being one of the constituents responsible for their antidepressant efficacy [16]. Transcriptomic analyses detected a unique upregulation of hippocampal PACAP expression post Yueju (unpublished).

However, it has not been evaluated whether the antidepressant effect of crocin is related to PACAP. In this study, we established a chronic unpredictable mild stress (CUMS) model of mice and corticosterone (CORT) model of PC12 cell to investigate the antidepressant effect of crocin and its related mechanism.

## 2. Materials and Methods

### 2.1. Animals

Male Balb/cJ mice (18-24 g, 8-10 weeks of age) were obtained from Jiangning Qinglongshan Animal Cultivation Farm (Nanjing, China, SCXK2017-0001) and housed under standard laboratory conditions. The mice were kept in cages under a 24 h day and night cycle light environment, 50 ± 10% humidity, and a temperature of 24 ± 1°C with free access to water and food. They were acclimatized for 1 week before the CUMS procedures were initiated. All animal work was conducted in the animal center of Nanjing University of Chinese Medicine and carried out in accordance with the principles of the Basel Declaration and recommendations of the International Association of Veterinary Editors guidelines for the care and use of laboratory animals in Nanjing University of Chinese Medicine. The protocol was approved by the Experimental Animal Ethics Committee of Nanjing University of Chinese Medicine (experimental animal ethics batch number: 201906A007).

### 2.2. Preparation and Identification of *β*-D-Gentiobiosyl Crocetin

The fruit of *Gardenia jasminoides* Ellis (5 kg) was refluxed with 50% aqueous ethanol (EtOH) for 2 h at 100-110°C three times. After solvent removal, the combined residues were separated on a macroporous resin column (2540 g, 20-40 mesh) with gradient (EtOH/H_2_O, 0 : 100⟶EtOH/H2O, 20 : 80⟶EtOH/H2O, 50 : 50) to yield 3 fractions (Fr.1-Fr.3). Fr.3 (474 g) was further subjected to a Sephadex LH-20 column eluted with EtOH/H_2_O (50 : 50) to afford total crocin. Finally, *β*-D-Gentiobiosyl Crocetin was obtained by RP-18 silica gel column chromatography (Wanqing Chemical Glassware & Instrument Co., Ltd., Nanjing, China) using MeCN-H2O (30 :200970) from total crocin.

Identification of *β*-D-Gentiobiosyl Crocetin is as follows: HR-ESI-MS m/z: 675.2620 [M+Na]+(calculated for C32H44O14Na [M+Na] +, 675.2629). 1H-NMR (400 MHz, DMSO-d6) *δ*: 7.36 (1H, H-10), 7.20 (1H, H-10′), 6.84 (1H, H-15′), 6.82 (1H, H-15), 6.78 (1H, H-12), 6.71 (1H, H-11′), 6.65 (1H, H-11), 6.63 (1H, H-12′), 6.51 (1H, H-14), 6.50 (1H, H-14′), 5.42 (2H, H-1′), 1.99 (6H, H-19, 19′), 1.97 (3H, H-20), 1.92 (3H, H-20′). The above data are in agreement with the literature [17].

### 2.3. Model and Treatment

The CUMS procedure was performed as described earlier [18] with minor modifications. The mice were assigned randomly to four groups (*n* = 10 each): control (sodium chloride 0.9%), CUMS, CUMS plus crocin 30 mg/kg (intragastric administration, ig), and CUMS plus fluoxetine (Flx) 20 mg/kg (intraperitoneal injection, ip). From the third week, crocin and Flx were administered once daily until the CUMS paradigm end (Figure 1(a)). Flx (54910-89-3) was purchased from TCI (Shanghai, China).

### 2.4. Behavioral Evaluation

All mice underwent depression-like behavioral tests after CUMS. The protocol followed in sequence: open-field test (OFT), tail suspension test (TST), forced swimming test (FST), sucrose preference test (SPT), and novelty-suppressed feeding (NSF). The behavior tests were carried out according to previous literature of our group [18]. After the behavioral experiments were over, mice were sacrificed by decapitation.

### 2.5. Cells Culture

PC12 cells were seeded in a 96-well plate at a density of 5 × 10^4^cells per well and incubated for 24 h. The cells were pretreated with gradient concentrations of crocin (12.5, 25, and 50 *μ*M) for 1 h and then treated with CORT (200 *μ*M) for 24 h. CORT (#C104537) was provided by Aladdin (Shanghai, China). Cell viability was assessed by 3-(4,5-Dimethylthiazol-2-yl)-2,5-diphenyl tetrazolium bromide (MTT) assay obtained from Biofrox (#298-93-1, Germany). For Hoechst fluorescent staining, the cells were fixed with 4% paraformaldehyde at room temperature for 30 min, followed by staining with Hoechst 33258 solution at 37°C for 10 min. The cells were then washed with phosphate buffer saline (PBS), and images were obtained with a fluorescence microscope. Hoechst 33258 (FXP138-1000) was purchased from Sizhengbai Biotechnology Co., Ltd. (Beijing, China).

### 2.6. Transfection

PACAP RNA interference (RNAi) was provided by Nanjing KeyGen Biotech. Co., Ltd. (Nanjing, China). After anesthetized, the mice were place in a stereotactic apparatus. Lentivirus for PACAP siRNA with a Hamilton syringe was injected into the prefrontal cortex. At least 7 days of recovery were required before sample collection. PC12 cells were transfected with PACAP RNAi or negative control RNAi for 5 h via lentivirus with the Opti-MEM Reduced Serum Medium. The medium was then replaced with the regular culture medium containing serum, and the cells were cultured for 48 h. Next, the cells were exposed to CORT (200 *μ*M) with or without crocin (25 *μ*M). Finally, we used western blotting analysis to evaluate the efficiency of PACAP RNAi (Figure 2).

### 2.7. Western Blotting

The PC12 cells were homogenized and lysed in ice-cold radio immunoprecipitation assay (RIPA) solution. Antibodies were obtained from commercial sources: p-ERK (4376) [19], EKR (9102), CREB (9197), and p-CREB (9198) [20] were from Cell Signaling Technology (CST, USA); PACAP (0190R) was from Beijing Biosynthesis Biotechnology Co., Ltd. (Beijing, China), and PACAP (sc-166180) was from Santa Cruz [21–23]; Tubulin (10094-1-AP) [24] was from Proteintech (Chicago, USA).

### 2.8. Statistical Analysis

All data were expressed as mean ± SEM, and differences between groups were analyzed using one-way ANOVA and *T*-test. *P* < 0.05 was considered statistically significant. All data in the figures were obtained using GraphPad Prism 5 statistical software.

## 3. Results

### 3.1. Crocin Reversed the Decreases of Body Weight and Elevation of Serum CORT

As shown in Figures 1(b) and 1(c), the body weights of the mice in each group had no differences at the beginning. Over the 3-week and 7-week modeling, CUMS reduced the body weight gain of mice (*P* < 0.01, *P* < 0.01), crocin significantly increased the body weight after 7 weeks compared with CUMS group (*P* < 0.01), but Flx did not.

Hypothalamic-pituitary-adrenal (HPA) axis is a major neuroendocrine system closely associated with stress induced depression; the activity of which was quantified with the determination of the serum level of CORT. The level of CORT was higher in the CUMS groups than that in the saline group (*P* < 0.01), but crocin and Flx reversed the elevation of serum CORT (*P* < 0.01, *P* < 0.01) (Figure 1(d)). These results indicated that crocin reversed the growth of body weight and attenuated CUMS-induced hyperactivity of HPA axis.

### 3.2. Crocin Reversed CUMS-Induced Depression-Related Behavior

With the SPT, reflecting anhedonia, the sucrose consumption rate in the CUMS group was obviously lower than that in the saline group (*P* < 0.01). After crocin treatment, the decrease of the percentage of sucrose preference was reversed (*P* < 0.01) (Figure 3(a)). The TST and the FST results reflected the behavioral despair of the mice. We found that the immobility time of the CUMS group was extended remarkably compared with the saline group (*P* < 0.01, *P* < 0.01), while crocin shortened the immobility time (*P* < 0.01, *P* < 0.01) (Figures 3(b) and 3(c)). The NSF test showed that CUMS had reduced food consumption (Figure 3(d)) and increased feeding latency significantly (*P* < 0.01, *P* < 0.01) (Figure 3(e)), while crocin treatment reversed these phenomena (*P* < 0.01, *P* < 0.01). These effects of crocin were similar to those of the classic antidepressant fluoxetine. The OFT evaluates locomotor activity, which was not affected by CUMS stimulation or crocin and fluoxetine administration (Figures 3(f) and 3(g)).

### 3.3. Crocin Relieved Corticosterone-Induced PC12 Injury

To validate the antidepressant effects of crocin, we established a corticosterone model in PC12 cells. The cells were administrated with gradient concentrations of crocin (12.5, 25, and 50 *μ*M) for 1 h, then CORT (200 *μ*M) for 24 h. Data from Hoechst 33258 staining are shown in Figure 4(a). The PC12 cells in the control group had large nuclei, complete and regular morphology, and uniform fluorescence distribution. However, after CORT (200 *μ*M) treatment, the number of nuclei was significantly reduced, with irregular morphology, condensed chromatin, uneven fluorescence distribution, and nuclear fragmentation. These were typical characteristics of apoptosis. MTT results showed that the cellular viability of PC12 cells was 61.4% in the CORT group (*P* < 0.01), while increased to 95.2%, 102.2%, and 106.2% (*P* < 0.01, *P* < 0.01, and *P* < 0.01) after crocin treatment (12.5, 25, and 50 *μ*M) (Figure 4(b)); hence, we chose 12.5 *μ*M crocin for the later experiment. These results indicated that crocin has a neuroprotective effect against CORT-induced damage.

### 3.4. Crocin Increased PACAP Expression and Phosphorylation of CREB and ERK in the Corticosterone Cell Model

To explore the antidepressant mechanism of crocin, we analyzed the expression of PACAP and associated signaling pathways. Compared with the control group, the expression of PACAP was significantly decreased in the CORT group (*P* < 0.01) but reversed by crocin (*P* < 0.01). Furthermore, CORT inhibited the phosphorylation of CREB and ERK (*P* < 0.01, *P* < 0.05), but this effect was suppressed by crocin (*P* < 0.01, *P* < 0.05) (Figures 4(c)–4(f)).

### 3.5. PACAP Was Involved in the Neuroprotective Effects of the Crocin In Vitro Model of Depression

To confirm whether PACAP was responsible for the antidepressant effect of crocin, we downregulated PACAP expression using RNAi based on the PC12 cells. 293 T cells and PC12 cells were transfected with control RNAi and PACAP RNAi for 5 h. After resting 48 h, we observed that most of the cells emitted fluorescence with PACAP RNAi but not control RNAi, indicating successful transfection (Figure 5(a)). Compared with the control group, PACAP RNAi transfection was shown to significantly reduce PACAP expression to 54.2% (*P* < 0.01) (Figures 5(b) and 5(c)). Finally, we used PACAP RNAi to transfect PC12 cells and treated the cells with crocin and CORT. Hoechst staining and MTT assay results revealed that CORT reduced the viability of PC12 cells compared with the control group obviously (*P* < 0.01) (Figures 5(d)–5(f)), which was reversed by crocin (*P* < 0.01). However, PACAP RNAi reduced PC12 cell viability noticeably. Therefore, transfection of PACAP RNAi significantly abolished the neuroprotective effects of crocin in the CORT cell model. Thus, it could be extrapolated that PACAP may be involved in the antidepressant effect of crocin.

## 4. Discussion

Major depression is a common illness that severely limits psychosocial functioning and diminishes quality of life. Studies have shown that depression is expected to be the second most common disease after cardiovascular disease [25]. However, our knowledge of the pathophysiology of depression is incomplete, which prevents us from developing more effective treatments so far. Recent studies have reported that traditional Chinese medicine (TCM) has significant clinical effects in the prevention and treatment of depression [26]. In the present study, we purified crocin from the fruit of *Gardenia jasminoides* Ellis and study the antidepressant effect and mechanism of crocin. We found that crocin reversed the decrease of body weight and elevation of serum CORT. Further, crocin increased food consumption and decreased the feeding latency, increased the sucrose consumption rate, and reduced the immobility time in TST and FST assessments of CUMS model mice. These indicated that crocin could moderate the observed depression-like behavior the same as fluoxetine in the CUMS model. In addition, crocin reduced apoptosis in the CORT model in PC12 cells, as demonstrated by Hoechst staining and MTT assay. Meanwhile, crocin increased the expression of PACAP and phosphorylation of CREB and ERK. Transfection of PACAP RNAi significantly abolished the protective effects of crocin in the CORT cell model. These suggested that PACAP was involved in the neuroprotective effects of crocin.

As a consequence of CUMS, reduction of body weight gain and elevation of serum CORT were observed, indicating alterations in adrenal cortex function. In addition, the weight of adrenal and thymus demonstrated an inhibition of the immune system after long-term stress [27]. Our results indicated that crocin markedly ameliorated the function of the HPA axis and potentially affected the adrenal and thymus glands. Previous studies have confirmed that crocin decreased dietary intake and reduced the appetite of patients with coronary artery disease [28] and the obese Wistar rat [29], which has antiobesity and anorectic effects. These studies did not describe the effects of crocin on normal people or normal animals. Actually, we found that crocin alone did not affect the behavior of mice in NSF and SPT in our previous study. However, in the specific CUMS model, crocin increased the intake of food and sucrose and improved the appetite of mice with depression.

The ERK-CREB pathway plays a key role in the treatment of depression [30, 31]. It can be activated by many antidepressant drugs, including paeoniflorin [32] and memantine [33]. Gardenia yellow pigment (GYP) is a class of compounds with a crocin structure. GYP could activate ERK, CREB and their downstream effectors, which were thought to be response to neuronal survival and neuroplasticity, thereby exerting rapid antidepressant effects in learned helplessness paradigm [16]. In our experiment, crocin significantly increased ERK and CREB phosphorylation, while the expression of total ERK and CREB proteins did not change. This suggested that the antidepressant effect of crocin was through increased phosphorylation of ERK and CREB. PACAP, a potent neuropeptide, binds to G-protein coupled receptor (GPCR) isoforms and activates downstream signaling pathways including the protein kinase A- (PKA-) CREB pathway [10, 30]. Over the past ten years, increasing evidences supported that PACAP might play a modulatory role in stress-related mood disorders and stress adaptation [34, 35]. Human genetic variants of PACAP or its receptor were found to be associated with depression and posttraumatic stress disorder (PTSD), particularly in females [36]. However, there were also studies suggesting that PACAP administration had anxiogenic and depressive effects [37], and PACAP deficiency seemed to be protective against social defeat [38]. It has been shown that different phenotypes of PACAP KO mice depend on genetic background. PACAP KO mice (F1: C57BL/6J × 129SvEv) exhibited increased locomotor activity in a novel environment and abnormal anxiety-like behavior but showed slightly decreased depression-like behavior [39]. CORT elevation and weight loss following 7-day chronic restraint stress are severely blunted in PACAP-deficient mice (C57BL/6N) [40]. PACAP-deficient mice on CD1 background were shown to have depression-like phenotype [41]. Our research applied RNA interference to confirm that PACAP elevation had an antidepressant effect by activating the ERK-CREB signaling pathway. Furthermore, crocin upregulated endogenous PACAP to activate ERK and CREB and improved depressor-like behaviors in CUMS mice.

The present study supports the hypothesis that stress inhibits the expression of PACAP, thereby inhibiting the phosphorylation of its downstream ERK and CREB, and then reduces the translation of synaptic plasticity proteins, finally leading to depressed-like behaviors. Crocin can activate ERK and CREB signaling pathways via upregulating endogenous PACAP, then enhance synaptic plasticity and improve neuron survival, and play an antidepressant role in the mice CUMS model and the corticosterone cell model (Figure 6). It is thus conceivable that PACAP will be an important target for antidepressant treatment. In addition, we believe that TCM has its unique advantages in treating depression. However, TCM has multiple targets and approaches, and the research on TCM treatment of depression should be further standardized to better guide clinical practice.

## Figures and Tables

**Figure 1:** Crocin reversed the decreases of body weight and elevation of serum CORT. (a) Schematic diagram of the experimental process of chronic unpredictable mild stress (CUMS) program and treatments. (b) Weight change in 0-7 weeks' model process. From the first week to 7th week: two-way ANOVA, *F* (2, 57) = 5.819, *P* = 0.005; *F* (2, 57) = 22.24, *P* < 0.0001; F (1, 57) = 16.58, *P* = 0.0001. All data are expressed as mean ± SEM. ∗*P* < 0.05, ∗∗*P* < 0.01 compared with the control group. (c, d) The weight and levels of CORT change. ANOVA, *F* (3, 28) = 6.010, *P* = 0.0027; *F* (3, 28) = 20.67, *P* < 0.0001. All data are expressed as mean ± SEM. ∗P < 0.05, ∗∗*P* < 0.01 versus saline; ^#^*P* < 0.05, ^##^*P* < 0.01 versus CUMS.

**Figure 2:** Western blotting analysis of the expression of PACAP. Representative diagram for the sites of the prefrontal cortex transfection of PACAP RNAi or scramble control sequence (SCR). *T*-test, ^∗^*P* < 0.05 versus SCR group, *n* = 3.

**Figure 3:** Crocin recovered CUMS-induced depression-related behavior. (a) The sucrose preference test. ANOVA, *F* (3, 26) = 38.07, *P* < 0.0001. (b, c) The immobility time in TST and FST. ANOVA, *F* (3, 26) = 56.74, *P* < 0.0001; ANOVA, *F* (3, 26) = 16.72, *P* < 0.0001. (d, e) The food consumption and feeding latency in NSF. ANOVA, *F* (3, 25) = 37.15, *P* < 0.0001; ANOVA, *F* (3, 26) = 33.55, *P* < 0.0001. (f, g) The total distance and time in center in OFT. ANOVA, *F* (3, 22) = 1.019, *P* = 0.4031; ANOVA, *F* (3, 26) = 1.238, *P* = 0.3162. All data are expressed as mean ± SEM. ∗*P* < 0.05, ^∗∗^*P* < 0.01 versus saline; ^#^*P* < 0.05, ^##^*P* < 0.01 versus CUMS.

**Figure 4:** Crocin relieved corticosterone induced PC12 injury by regulating PACAP-mediated ERK and CREB signaling pathways. (a) Hoechst 33258 staining and observation of PC12 cells with fluorescence microscope. (b) Effect of crocin in cell viability using MTT assay. ANOVA, *F* (5, 30) = 24.97, *P* < 0.0001. (c-f) PACAP, ERK, and CREB were analyzed by immunoblotting. ANOVA, *F* (3, 8) = 23.77, *P* = 0.0002; ANOVA, *F* (3, 10) = 3.265, *P* = 0.0676; ANOVA, *F* (3, 10) = 15.86, *P* = 0.0004. Data are expressed as mean ± SEM (*n* = 3). ^∗^*P* < 0.05 and ^∗∗^*P* < 0.01 versus the control group; ^#^*P* < 0.05 and ^##^*P* < 0.01 versus CORT group.

**Figure 5:** PACAP was involved in the neuroprotective effects of crocin in the CORT model of PC12 cells. (a) Knockdown of PACAP with PACAP siRNA. The cells were observed under the fluorescence microscope. (b-c) Western blotting analysis of the expression of PACAP after transfection with PACAP siRNA. *T*-test, *n* = 5, *P* < 0.01. (d) Hoechst33258 staining and observation of PC12 cells with fluorescence microscope after transfection with PACAP siRNA and crocin. (e) Effects of crocin in cell viability of PC12 cell after transfection with PACAP siRNA. ANOVA, *F* (3, 24) = 75.75, *P* < 0.0001. ^∗^*P* < 0.05 and ^∗∗^*P* < 0.01 versus control group; ^#^*P* < 0.05 and ^##^*P* < 0.01 versus CORT group, ^$^*P* < 0.05 and ^$$^*P* < 0.01 versus CORT+crocin group.

**Figure 6:** A schematic illustration of the proposed mechanism for the neuroprotective effect of crocin in depression. Stress inhibits the expression of PACAP, thereby inhibiting the phosphorylation of its downstream ERK and CREB, and then reduces the translation of synaptic plasticity proteins, finally leading to depressed-like behaviors. Crocin can activate ERK and CREB signaling pathways via upregulating endogenous PACAP, then enhance synaptic plasticity and improve neuron survival, and play an antidepressant role in mice CUMS model and corticosterone cell model.

## Data Availability

The data used to support the findings of this study are available from the corresponding author upon request.
